The article "Abnormal brain structure in atopic dermatitis: Evidence from Mendelian randomization study" was retracted in 2025. Reasons: unreliable data; unreliable results or conclusions; concerns about the peer review.

# Abnormal brain structure in atopic dermatitis: Evidence from Mendelian randomization study

**DOI:** 10.1111/srt.13515

**Published:** 2023-11-16

**Authors:** Yue Chen, Liqian Cui, Hao Li, Aili Gao

**Affiliations:** ^1^ Department of Dermatology Guangzhou Institute of Dermatology Guangzhou Guangdong China; ^2^ Department of Neurology The First Affiliated Hospital Sun Yat‐sen University Guangzhou China; ^3^ Department of Neurology Donders Center for Medical Neurosciences Radboud University Medical Center Nijmegen The Netherlands

**Keywords:** atopic dermatitis, brain cortical structure, causal effect, Mendelian randomization

## Abstract

**Background:**

Structural abnormalities in the brain of patients with atopic dermatitis (AD) have been reported; however, the cause has not been determined yet. Herein, we used Mendelian randomization (MR) to reveal the causal effect of AD on brain structure.

**Methods:**

This study utilized summary statistics from genome‐wide association studies (GWASs) to investigate a collection of cerebral structural measures, encompassing cortical thickness (CT), cortical surface area (CA), and subcortical volumes in T1 images. A comprehensive GWAS meta‐analysis identified a total of 20 independent single nucleotide polymorphisms linked to AD, surpassing the genome‐wide significance threshold (*p* < 5 × 10⁻⁸). MR estimates were aggregated through the application of the inverse variance weighted method. Additional complementary analyses (i.e., MR‐Egger and weighted median approaches) were conducted to further assess the robustness of the obtained results. Sensitivity analysis and multivariate MR (MVMR) while adjusting for brain structural changes risk factors (i.e., depression and anxiety) were performed to assess the reliability and stability of observed causality.

**Results:**

Genetically determined AD exhibited a causal link with reduced caudate volumes (IVW‐MR: β = ‐0.186, *p* = 0.001, *p*‐corrected = 0.009). Furthermore, we identified potential causal associations between AD and reduced CT in the cingulate region (posterior cingulate, IVW‐MR: β = ‐0.065, *p* = 0.018, *p*‐corrected = 0.551; isthmus cingulate, IVW‐MR: β = ‐0.086, *p* = 0.003, *p*‐corrected = 0.188), as well as abnormal cortical surface area (CA) in the supramarginal (IVW‐MR: β = ‐0.047, *p* = 0.044, *p*‐corrected = 0.714) and isthmus cingulate (IVW‐MR: β = 0.053, *p* = 0.018, *p*‐corrected = 0.714). Additional supplementary analyses yielded consistent outcomes. There was no evidence of horizontal pleiotropy. MVMR analysis showed that the causal effects of AD on abnormal brain structure remained significant while adjusting for depression and anxiety.

The article "Abnormal brain structure in atopic dermatitis: Evidence from Mendelian randomization study" was retracted in 2025. Reasons: unreliable data; unreliable results or conclusions; concerns about the peer review.

**Conclusion:**

This MR study provided suggestive evidence that decreased caudate nucleus, posterior cingulate cortex, isthmus cingulate cortex and supramarginal gyrus are suggestively associated with higher AD risk. Future investigation into the brain regions is recommended, which helps to clarify the underlying mechanisms and point to new therapies against AD.

## 1 INTRODUCTION

Atopic dermatitis (AD), also known as eczema, is a persistent inflammatory skin disorder affecting approximately 25% of children and between 5–10% of adults globally.^1^, ^2^ One of the main features of AD is severe pruritus, which can lead to recurrent eczematous skin rashes. Pruritus‐related disturbances, such as sleep disruption and decreased work productivity, significantly impact patients' quality of life.^3^ However, the pathogenesis of AD is multifactorial, complex, and poorly understood, leading to limited treatment options. In recent years, evidence has emerged linking AD with neuropsychological conditions, including abnormal brain function. Specifically, one study found that AD participants with an itch state had increased neuronal activity in certain brain regions, such as the insula, striatum, and prefrontal cortex, as measured by resting‐state functional MRI.^4^ Another study, which used arterial spin labeling (ASL) to measure cerebral blood perfusion, reported an increase in blood supply in similar brain regions.^5^ In addition, a recent study using Electroencephalography (EEG) to measure brain activity also reported abnormally high activity in the right frontal lobe in ad patients.^6^ This can be attributed to two primary factors. Firstly, AD is characterized by a vicious cycle of itching and scratching, potentially linked to an intracranial reward loop. Secondly, AD often co‐occurs with psychiatric conditions, such as depression and/or anxiety. These neuropsychological conditions may also contribute to the exacerbation of AD. Alterations in brain structure and function may also drive this cycle. However, these previous findings have heavily relied on cross‐sectional observational studies, which inherently constrain the ability to establish causation. Furthermore, prior studies have primarily focused on the functional abnormalities in the cerebral aspect of AD, while the structural changes, which are considered the underpinnings of abnormal functional activities, have received limited attention.

To overcome these limitations, we employed Mendelian randomization (MR) analysis, an emerging approach for causal inferences.^7^ Based on the premise of random genetic variant assortment during meiosis, the MR approach leverages these genetic variations linked to phenotype as instrumental variables (IVs) to deduce the association between exposures (i.e., AD in the present study) and outcomes (i.e., brain structure in the present study).^8^ As genetic variants are randomly assigned at conception, before the onset of disease, MR analysis is well‐positioned to address confounding factors and reverse causality, hence identifying potential causal associations between the exposure and the outcomes.^9^  In this study, we aimed to determine the potential causal relationship between AD and abnormal brain structure, providing a theoretical basis for understanding the itch in AD. To this end, we performed two sample MR analyses between the AD and the cerebral structural measures, including the cortical thickness (CT), CA, and subcortical volumes in T1 images, using the large‐scale genome‐wide association study (GWAS) data.

The article "Abnormal brain structure in atopic dermatitis: Evidence from Mendelian randomization study" was retracted in 2025. Reasons: unreliable data; unreliable results or conclusions; concerns about the peer review.

## 2 MATERIALS AND METHODS

### 2.1 Study design

The present MR analysis between AD and cerebral structures was performed based on Strengthening the Reporting of Observational Studies in Epidemiology using Mendelian Randomization (STROBEMR) statement, as shown in Figure 1.^10^ Analyses followed three predominant assumptions: (1) IVs should be highly correlated with the exposure elements; (2) IVs should be independent of confounding factors; (3) IVs should affect the outcome solely through exposure.^11^ Single nucleotide polymorphisms (SNPs) were selected as IVs due to their random allocation and lower susceptibility to confounding or reverse causation.^12^

**FIGURE 1:** Study design flowchart of the Mendelian randomization study.

### 2.2 Data source and IVs selection

The SNP dataset for AD was obtained from the IEU database (https://gwas.mrcieu.ac.uk/, ID: finn‐b‐L12_ATOPIC). It comprised 7024 AD cases and 198,740 controls of European ancestry. A total of 20 SNPs were identified as potential IVs for AD based on a significance threshold of *p* < 5 × 10^−8^ and a linkage disequilibrium threshold of r^2^ = 0.001 within a 10,000 kb genomic window.

The SNP dataset for cerebral structural measures, including CT, CA, and subcortical volumes, were obtained from a previously published GWAS study.^13^ This study explored the genetic associations of cerebral structural measures in a sample of 8428 individuals. Cortical measures, namely CT and CA, for each cortical region, were extracted using the Desikan–Killiany–Tourville (DKT) atlas, which parcellates the cortex into 31 distinct.^9^ Subcortical volumes, encompassing the caudate, thalamus, pallidum, putamen, amygdala, hippocampus, and accumbens, were also calculated. In line with the IVs selection for AD, SNPs with a significance threshold of *p* < 5 × 10^−8^ and a linkage disequilibrium threshold of r^2^ = 0.001 were identified as potential IVs.

The article "Abnormal brain structure in atopic dermatitis: Evidence from Mendelian randomization study" was retracted in 2025. Reasons: unreliable data; unreliable results or conclusions; concerns about the peer review.

Finally, we utilized PhenoScanner, an online tool available at www.phenoscanner.medschl.cam.ac.uk, to identify the aforementioned potential IVs as well as confounding factors. Conditions like inflammatory bowel disease and alopecia areata, along with medical issues such as endocrine or autoimmune diseases, were considered as exclusion criteria due to their potential to affect the study's integrity. SNPs correlating with potential confounders were eliminated from our set of IVs.^14^

### 2.3 Statistical analyses

To begin with, we employed the MR‐PRESSO (Mendelian Randomization Pleiotropy REsidual Sum and Outlier) test to identify the outlier SNPs. If an SNP was identified as an outlier (determined by an MR‐PRESSO global test *p*‐value < 0.05, indicating potential horizontal pleiotropy), it was subsequently excluded from the analysis.^15^ Next, the inverse‐variance weighting‐based MR (IVW‐MR) analysis was employed to estimate the causal association between AD and each cerebral structure measure (i.e., regional CT, SA and subcortical volumes).^16^ When a significant association between the cerebral structure measure and AD was identified, subsequent MR analyses using both MR‐Egger and weighted median methods were performed to validate the consistency in the direction of the estimates using three methods. IVW‐MR was chosen as the primary analysis due to its high accuracy and power in the estimation, whereas MR‐Egger and weighted median served as supplementary analyses as they provide more robust but less powerful estimations.^17^ Lastly, to ensure the robustness of our findings, a series of sensitivity analyses were conducted. The intercept test in MR‐Egger regression was employed to test directional pleiotropy, a condition arising when genetic variation significantly impacts outcomes through non‐exposure pathways; the Cochrane's Q test was employed to identify potential horizontal pleiotropy, which occurs when genetic variants affect the outcome through alternative pathways other than the exposure of interest; the leave‐one‐out analysis was employed to assess the influence of individual SNPs on the MR estimates, ensuring that no single SNP disproportionately impacted the results; the funnel plot was employed to assess the potential directional pleiotropy.^18^ Additionally, we performed multivariate Mendelian randomization (MVMR) analyses to reassess the observed causal association between AD and MRI‐confirmed structural abnormalities in the brain, while accounting for potential confounders such as depression and anxiety. Summary‐level data for these confounders were obtained from the MRC IEU Open GWAS Project of the UK Biobank, which included 113,769 depression cases versus 208,811 controls (ebi‐a‐GCST005902) and 53,414 anxiety cases versus 407,288 controls (ukb‐b‐18336).^19^ The flowchart of MR analysis is shown in Figure 1.

The article "Abnormal brain structure in atopic dermatitis: Evidence from Mendelian randomization study" was retracted in 2025. Reasons: unreliable data; unreliable results or conclusions; concerns about the peer review.

All analyses were performed using the ‘TwoSampleMR’ package within R (version 4.5.2). *p*‐Values were corrected for multiple comparisons using the *Benjamini‐Hochberg* based false discovery rate (FDR) approach. The significant level was set at a two‐tailed *p*‐*corrected* value < 0.05. The *p‐corrected* value > 0.05, but the *p*‐value < 0.05 was considered a borderline significance.

## 3 RESULT

A total of 20 SNPs were identified as candidate IVs for AD. All of the SNPs were inherited independently and without LD. Through phenoscanner, we found four SNPs correlated with potential confounding factors: rs6543132 and rs10208309 relate with Crohn's disease, rs28371176 relates with inflammatory bowel disease, and rs2236295 relates with alopecia areata. The four SNPs were discarded, resulting final 15 SNPs being employed as IVs for AD in the analysis (Table S2).

### 3.1 AD and cortical thickness

We found a borderline significant association between AD and the decreased CT in the posterior cingulate (IVW‐MR: β = −0.065, *p* = 0.018, *p‐corrected =* 0.551) and isthmus cingulate regions (IVW‐MR: β = −0.086, *p* = 0.003, *p‐corrected =* 0.188) (Figure 2, Table S3).

**FIGURE 2:** Association between genetically determined brain structural alterations and AD risks. This result also survived FDR correction for multiple comparisons (corrected significance threshold *p* = 0.05). AD, atopic dermatitis; Cl, confidence interval; OR, odds ratio; SNP, single nucleotide polymorphism.

### 3.2 AD and CA

We found a borderline significant association between AD and the decreased SA in the supramarginal region (IVW‐MR: β = −0.047, *p* = 0.044, *p*‐corrected = 0.714) and the increased SA in the isthmus cingulate regions (IVW‐MR: β = 0.053, *p* = 0.018, *p*‐corrected = 0.714) (Figure 2, Table S3). The results estimated by MR Egger and weighted median methods were in the same direction (Table S3).

### 3.3 AD and subcortical volumes

We found that AD was associated with decreased volumes in caudate (β = −0.186, *p* = 0.001, *p*‐corrected = 0.009, Figure 2, Table S3). The results estimated by MR Egger and weighted median methods showed a similar result/or were in the same direction (Table S3).  The scatter plots of MR analyses for AD in abnormal brain structure are exhibited in Figure 3.

**FIGURE 3:** Scatter plots of MR analyses for AD in abnormal brain structure. AD, atopic dermatitis, MR, Mendelian randomization.

The article "Abnormal brain structure in atopic dermatitis: Evidence from Mendelian randomization study" was retracted in 2025. Reasons: unreliable data; unreliable results or conclusions; concerns about the peer review.

### 3.4 Sensitivity analysis

The above MR analyses between AD and cerebral structural abnormalities (i.e., CT in the posterior cingulate and isthmus cingulate regions, SA in the supramarginal and isthmus cingulate regions, and volumes in the caudate), yielded results where both the intercept test in MR‐Egger regression and Cochrane's Q test indicated the absence of directional or horizontal pleiotropy (Table S4). Furthermore, MR‐PRESSSO did not reveal any outliers, and the analysis using the leave‐one‐out plot, along with the presentation of funnel plots and scatter plots (Supplementary Figure S1–S19), confirmed the absence of outliers. Our analyses demonstrated that the estimates remained unbiased by individual SNPs, suggesting the robustness of the estimates.

### 3.5 Multivariable Mendelian randomization

To confirm the observed causal effects of AD on brain structure while anxiety and depression exist as additional exposure variables, MVMR analysis was performed. The details of these IVs are shown in the supplementary material. The results of MVMR showed that the causal effects of AD on brain structure remained significant while adjusting for vascular risk factors (Table S5).

## 4 DISCUSSION

In the present study, we leveraged the GWAS data of AD and various cerebral structural phenotypes and thereby performed MR analyses between AD and brain imaging phenotypes. To the best of our knowledge, this is the first study addressing the association between AD and cerebral structural abnormalities. Our findings suggested a casual association between AD and reduced caudate volumes and the potential causal associations between AD and decreased CT in the cingulate, as well as abnormal CA in the supramarginal and isthmus cingulate. Moreover, these associations remained consistent in MVMR analyses while adjusting for depression and anxiety.

Our study suggested a causal association between AD and reduced caudate volume. This observation is consistent with prior fMRI studies on AD, which indicated abnormal neural activation and increased blood perfusion in the caudate relative to healthy controls when processing itch.^5^, ^20^ While the precise mechanism underlying the association between AD and cerebral abnormalities remains largely unknown, our results, in conjunction with similar findings from prior studies, indicate a significant involvement of dysfunction in the dopamine‐related reward system (particularly the caudate nucleus, a key component of the dopamine system) in AD. This dopamine‐related reward system is closely associated with the itch and scratch cycle. Continuous itching often triggers patients to scratch, providing temporary relief from the itch and a simultaneous release of dopamine.^21^ However, this action can exacerbate the skin's inflammatory response and perpetuate the chronic nature of the itch, thus establishing a vicious itch‐scratch cycle.^22^ Thus, interventions that target the dopaminergic system, particularly the caudate nucleus, may be crucial for disrupting this cycle, especially for patients with limited control over their scratching behavior.

The article "Abnormal brain structure in atopic dermatitis: Evidence from Mendelian randomization study" was retracted in 2025. Reasons: unreliable data; unreliable results or conclusions; concerns about the peer review.

We found a potential association between AD and decreased CT in the isthmus and posterior cingulate regions. This result aligns with previous studies that showed abnormal activation of the cingulate cortex in AD patients.^5^, ^6^, ^23^ The cingulate cortex is a densely connected and metabolically active region of the brain.^24^, ^25^ It is believed to play a pivotal role in pain perception and episodic memory retrieval.^26^, ^27^ Consequently, the observed structural atrophy and abnormal functional activation may be associated with the cognitive evaluation of itch stimuli and impulse control and/or scratching urges.^28^ Note that, we found that AD was potentially related to an increase in CA in the isthmus cingulate. This might be attributed to a compensatory enlargement of the cortical area in this region following a reduction in CT. Additionally, our study suggested a potential association between AD and decreased CA in supramarginal regions. This finding is consistent with one previous fMRI meta‐analysis which identified the supramarginal gyrus as the region of somatosensory processing for itch.^29^

Notably, since ad patients often have comorbid anxiety/depression, it is difficult to distinguish whether the brain abnormalities found in the ad are caused by pruritus/scratching ring or anxiety/depression.^30^ In this case, we further performed MVMR analysis and found that the previously observed brain structural abnormalities were still unchanged after adjustment for depression and anxiety. This evidence further supports that the nodal alterations in AD are primarily associated with itch‐scratch rather than comorbid anxiety/depression.

Our study has several strengths. To the best of our knowledge, this is the first study to investigate the associations between AD and brain structure through large‐scale GWAS data and MR analysis methods. We employed comprehensive and detailed brain imaging phenotypes (i.e., CT, CA and subcortical volumes across different regions), thereby enabling a detailed assessment of the cerebral structural abnormalities in AD. In addition, our methodology (MR analysis) leverages the random allocation of genetic variants associated with the exposure/outcome, enabling a rigorous investigation into their causal relationship while avoiding the bias introduced by confounding factors and the potential for reverse causality in observational studies. Lastly, we conducted several sensitivity analyses, including a pleiotropic‐robust approach, to ensure the validity of our estimated causal association.

The article "Abnormal brain structure in atopic dermatitis: Evidence from Mendelian randomization study" was retracted in 2025. Reasons: unreliable data; unreliable results or conclusions; concerns about the peer review.

Several limitations should be acknowledged. Firstly, the study did not differentiate between different severity levels of AD, which is a standard practice in clinical settings where AD is diagnosed based on scores such as SCORAD (Scoring Atopic Dermatitis).^31^, ^32^ This limitation stems from the fact that the study used a public database that did not provide information on the severity of AD. Consequently, the study was unable to examine the relationship between AD and brain structure in individuals with mild, moderate, or severe AD separately. Future studies should consider the severity of AD and explore its potential impact on the relationship between AD and brain structure to address this limitation. Moreover, the analysis was limited to a single sample of European ancestry, and thus, the results may not be generalizable to other populations. Finally, there is a possibility that exposure and outcome populations overlap, particularly in the UK biobank cohort, which may bias the results. Nevertheless, one recent study found that two‐sample MR can be more reliable than one‐sample MR.^33^

In conclusion, we provided suggestive evidence that decreased caudate nucleus, posterior cingulate cortex, isthmus cingulate cortex, and supramarginal gyrus are suggestively associated with higher AD risk. Future investigation into the brain regions is recommended, which helps to clarify the underlying mechanisms and point to new therapies against AD.

## CONFLICT OF INTEREST STATEMENT

The authors declare no conflict of interest.

## ETHICS APPROVAL

Ethics approval and consent to participate. This article contains human participants collected by several GWAS. All participants gave informed consent in all the corresponding original studies. Here, we only used the publicly available, large‐scale GWAS summary datasets, and not the individual‐level data. Hence, ethical approval was not sought.

## INFORMED CONSENT STATEMENT

Not applicable.

## Supporting information

Supporting Information

Supporting Information

## Data Availability

Availability of data and materials. All relevant data are within the paper. The authors confirm that all data underlying the findings are either fully available without restriction through consortia websites or may be made available from consortia upon request. All data analyzed during this study are included in this article.
